# Analysis of the Diagnostic Effect of EUS-RTE on Giant Cystic Tumours of the Oesophagus Based on Cluster Analysis

**DOI:** 10.1155/2021/1395826

**Published:** 2021-11-03

**Authors:** Huizhen Yang, Zhenghang Zhang, Yingbi He, Bin Tian, Xiaozhen Zhang, Yingying Hao, Shuang Lu, Yanhua Tian

**Affiliations:** ^1^Department of Endoscopy, The Second People's Hospital of Jiaozuo City, Jiaozuo, Henan 454003, China; ^2^The First Affiliated Hospital of Henan Polytechnic University, Jiaozuo, Henan 454003, China

## Abstract

This paper presents an in-depth analysis and study of the diagnostic effectiveness of EUS-RTE in giant cystic tumours of the oesophagus utilizing cluster analysis. A new form of interval data expression was designed based on the cluster analysis algorithm, as well as a new way of updating the cluster radius and cluster centre. Feature triads are defined, eliminating the need to access all historical data at the time of update. It also prevents the case of overfusion of clusters and outputting only one cluster. If there exist a very low number of clusters, the newly merged clusters are reclustered according to the density clustering method for the internal data objects based on the cluster segmentation so that the data objects in the same cluster have a high similarity as possible. All accumulated electronic files of oesophageal cancer cases were collected and comprehensively organized, and all clinical data of 129 eligible cases with a total of 356 consultations were screened in strict accordance with inclusion and exclusion criteria. A database of oesophageal cancer cases was established using Visual FoxPro software, and frequency distribution, cluster analysis, association rule, and chi-square test were used to focus on mining the association between symptoms, disease mechanisms, prescriptions, and medications. The results were analysed and summarized. Overall, the therapeutic efficacy and safety of the three groups of treatment modalities for gastric mesenchymal tumours were positive, and the preoperative endoscopic treatment modalities should be selected based on the EUS-RTE characteristics of the tumour, the site, and the operator's skill level in a comprehensive manner.

## 1. Introduction

Oesophageal cancer occurs in all five continents of the world. The wide distribution and concentration of oesophageal cancer are its characteristics. Oesophageal cancer is often widely distributed in a region and concentrated to form a high incidence area, and there are also low incidence areas in the high incidence area, showing the relationship between geography and the occurrence of oesophageal cancer. The incidence level of oesophageal cancer varies widely among different regions and populations, with rural areas having a higher incidence than urban areas [1]. The aetiology of oesophageal cancer is still unclear, and with the development of epidemiology, it is found that the incidence of oesophageal cancer involves multiple factors, each of which can play different roles due to differences in their exposure opportunities and dose intake caused by differences in geography, customs, and lifestyle behavioural habits, and the main prevalence factors may vary from region to region [2]. Adverse psychological factors such as the history of mental stimulation, frequent depression, and long-term mental depression have a close relationship with the occurrence of oesophageal cancer. Experiments show that adverse psychological factors can cause a series of adverse physiological changes through the combined effects of intermediary mechanisms such as the vegetative nervous system, endocrine system, neurotransmitters, and immune system, which can disrupt the “self-stability” of the immune system and cause disorders of the immune system, thus triggering the occurrence of cancer. Therefore, the significance of some factors should be further explored through cross-regional comparison or long-term monitoring and observation; the development of prevention and treatment measures for oesophageal cancer should also be based on local conditions [3]. The development of oesophageal cancer prevention and control measures should also be tailored to local conditions.

Data mining techniques not only help people to obtain and deeply apply the surface information of data from data warehouses but also obtain the implicit information of data and help people to determine the trend of future data changes. Clustering analysis is one of the main data mining techniques, which usually groups data objects according to some similarity measure and under certain criteria. There is always the problem of K-value selection and initial clustering centroid selection, and these problems can also affect the effect of clustering. In order to avoid these problems, we can choose another more practical clustering algorithm, the hierarchical clustering algorithm. After clustering, the data can be divided into sets with special meanings, and then the data can be analysed to get the implied information. Tumour treatment has entered a period of multidisciplinary, multipathway, and multimethod integrated treatment, which still cannot be cured. The recurrence rate of oesophageal cancer after surgery is high, and even for early lesions, the overall survival rate in the postoperative years is still very low; some patients have serious destruction of organ function and immunity during radiotherapy and chemotherapy, and the toxic side effects are strong and intolerable [4]. A more adapted comprehensive treatment is being explored, and TCM treatment is indispensable. TCM focuses on holistic concepts, and treatment is centred on humans rather than the tumour. The immune function of the body is regulated by mobilizing the patient's potential to participate in the regulation of the tumour or timely correction of too much or too little in the regulation and timely elimination of residual tumour cells. Reversing precancerous lesions will prolong or stop recurrence, improve the quality of life, and achieve the goal of survival with tumors.

At present, most clustering algorithms are oriented to static offline data with definite data size and scale. These algorithms firstly store all the data to be processed in memory and obtain the approximate optimal clustering results through multiple iterations. However, increasingly uncertain data are being generated from various industries, making uncertain data gradually become an important object for data mining, and it is an important issue to better obtain and apply valuable information from uncertain data for judgment and prediction. Uncertain data is different from general data from the beginning of generation, so it is necessary to extend the existing clustering algorithms for deterministic data to generate clustering algorithms that are truly applicable to uncertain data. The size of data is growing exponentially with the increasing volume of data, and what kind of representation and efficient storage should be used is a very important issue; secondly, the data objects are no longer single-dimensional but multidimensional. It considers the requirements of the characteristics of multidimensional data on mathematical models and related calculation methods.

## 2. Related Work

The clustering analysis technique is an integral part of the machine learning field and belongs to the unsupervised learning model [5]. In the era of big data, it is not practical to rely only on manual mining of the value behind the massive amount of information, and clustering is an effective data processing method that can help people discover some correlations within the data and even make predictions about future trends based on the existing data. In recent years, clustering analysis has played a key role in many fields [6]. Taking regional economic development as an example, by extracting representative economic indicators to cluster analysis of regional economic development, we can have clearer understanding of the status of economic development in different regions, to facilitate the formulation of measures to further promote good and rapid economic development. At the same time, cluster analysis is also applied in medical, chemical, computer vision, pattern recognition, and other fields, and its advantages cannot be ignored [7]. Lu et al. combined the minimum spanning tree principle with k-means to find a reasonable initial centre of clustering [8]. Malheiros combined a region-limited strategy with a k-means algorithm to achieve adaptive selection [9].

In rare patients with liquefied tissue within the tumour, ultrasound may suggest the presence of fluidic dark areas or cystic echogenicity. Currently, the main ancillary test for preoperative diagnosis of GIST patients is endoscopy [10]. The endoscopic appearance of the gastric mucosa is mainly oval hemispherical or bulbous, with a wide base in most cases and a smooth mucosal bulge with clear demarcation from the surrounding area. However, the endoscopic presentation of GIST is not very specific; therefore, it is difficult to distinguish GIST from other tumours by the microscopic features alone, and there are limitations of endoscopy for exophytic GIST because the lesions are often located in the submucosa, so it is difficult to obtain biopsies [11]. Ultrasound endoscopy can better compensate for the shortcomings of ordinary endoscopy, with the advantage of being able to distinguish between various layers of the gastric wall, as well as determine the origin of the mass lesion, that is, the specific layer and specific tissue structure of the gastric wall from which it originates and detect exophytic GIST, which is difficult to detect by ordinary endoscopy. In addition, ultrasound endoscopy can also determine the cystic solidity of the tumour by its echogenicity [12]. In addition, ultrasound endoscopy can also determine the cystic solidity of the tumour by its echogenicity, thus further differentiating it from some other gastric tumours [13]. However, the application of RECIST morphological criteria based only on the change of tumour size does not accurately reflect the effect of tumour treatment, and there are limitations in using it to evaluate the targeted treatment of gastrointestinal mesenchymal tumours [14]. The Choi criterion combines two indicators, tumour length and CT value change, and has been proved to have high application value in evaluating the efficacy of tumour treatment. However, tumour changes on imaging are often overestimated and sometimes do not coincide with pathological changes, so assessment of efficacy by imaging is controversial.

To retain the real-time online processing feature of the ECM algorithm, this paper designs a new way of updating cluster centres and cluster radii based on the ECM algorithm and MU-ECM algorithm and proposes an evolutionary clustering algorithm with adaptive interval width: MU-SAECM algorithm. To satisfy the property of scanning once, a feature triad is defined for each cluster, which makes the algorithm perform the radius and centroid update calculation only for the updated cluster radius and cluster centre once, satisfying the processing of each data based on reduced computation. New determination rules are added to the categorization to prevent changes occurring due to clustering from affecting the dissimilarity between classes. At the same time, to avoid the excessive fusion of clusters that can lead to a low number of clusters, the idea of density-based partial clustering is introduced to improve the accuracy by partitioning the relatively large clusters internally into several different clusters.

### 2.1. Cluster Analysis of EUS-RTE in Giant Cystic Tumours of the Oesophagus Designed for Diagnostic Effectiveness

#### 2.1.1. Analysis of EUS-RTE Algorithm for Cluster Analysis

Collaborative filtering technology is widely used in recommendation systems due to its advantages of simple operation and high recommendation efficiency, and it has become one of the most popular recommendation techniques in the field of personalized recommendation. The cold start problem mainly includes user cold start and item cold start. The user cold start is based on new users, and new users are a major challenge in the recommendation field. The situation is similar for new items in the system, which do not receive any feedback from users at the initial stage, so they are almost impossible to be recommended and in most cases are ignored [15]. The traditional collaborative filtering algorithm calculates similarity based on rating data to form the final recommendation, and the richer the data, the higher the accuracy of the recommendation, which directly affects user satisfaction. The number of items in the system is increasing, but the number of items faced by a single user is limited, and a few users can make valid ratings for items, so the ratings in the system mostly exist as null values which has a great impact on the accuracy of recommendations.

Collaborative filtering technology is based on a large amount of data information to provide users with reliable recommendations. With the rapid development of network technology, the number of users and products is increasing, and the corresponding amount of rating data is also increasing. The computation of various data needed to generate recommendations based on all data information in the whole recommendation system is large and time-consuming, which makes the recommendation efficiency low, the recommendation real-time poor, and the accuracy of the recommended results limited [16]. The division-based clustering first needs to specify the number of clusters *k*. Assuming that the sample contains *n* data objects, *k*< *n* needs to be satisfied, and then *k* initial centroids are selected from the data samples and iterated until the initial threshold is satisfied or the maximum number of iterations is reached so that the distance between data samples within the class is small and the similarity is high, and the distance between data between classes is large and the similarity is low. The most widely cited method is the k-means algorithm, which divides the data set into *k* disjoint clusters according to the specified *k*-values, with a small distance between data in the same cluster and high data similarity and a large distance between data in different clusters and low data similarity.

(1) $$\begin{array}{c} E=\frac{\sum_{i=1}^{k}\sum_{x\in c_{i}}{\left\|x\right\|}^{2}}{\sum_{i=1}^{k}\sum_{x\in c_{i}}{\left\|\mu_{i}\right\|}^{2}}. \end{array}$$

The distance measure between data is the core step of the clustering algorithm, which is necessary for clustering the data. When clustering, data with small distances are classified into the same class of clusters, and data with large distances are classified into different classes of clusters. The traditional user-based collaborative filtering technique mainly calculates the similarity between users based on their past behavioural data and then selects the nearest users for rating prediction and recommendation generation based on the similarity size. However, new users do not generate behavioural data that can be used for recommendations, and recommendations are hampered; at the same time, as user data and project data continue to grow, the scalability problem poses a growing challenge. At the same time, the soft clustering algorithm replaces the hard clustering algorithm, and the affiliation degree replaces the hard division of either/or, which is closer to real life. Secondly, based on the user's attribute data, we combine the improved clustering algorithm to cluster the users, so that new users can also be classified into the corresponding class clusters based on the attribute data information at the time of registration. Finally, the weighted similarity calculation of the similarity of user attributes is carried out in the clusters to which the user belongs, to improve the accuracy of user similarity calculation. At the same time, for new users with missing behavioural data, the nearest-neighbour selection and rating prediction can also be carried out based on the similarity of user attributes, to form recommendations and alleviate the drawbacks brought about by user cold start. At the same time, the selection of nearest-neighbour users in the cluster to which they belong reduces the scope of user search, reduces the amount of computation, and alleviates the disadvantages of recommendation scalability problems, as shown in Figure 1.

The digitized user attribute values are further normalized, and the normalization calculation is shown in

(2) $$\begin{array}{c} x^{*}=\frac{x-x_{\min}}{x_{\max}+x_{\min}}. \end{array}$$

Based on the normalized user attribute data for the calculation of user attribute similarity, the Euclidean distance is first selected for the initial calculation, which is shown in

(3) $$\begin{array}{c} \text{distance}=\sqrt{\sum_{i=1}^{n}{\left(x-\mu_{i}\right)}^{2}}. \end{array}$$

Based on the obtained Euclidean distance between users, the user attribute similarity is further calculated as shown in

(4) $$\begin{array}{c} {\text{sim}}_{d}\left(u,v\right)=\frac{1}{1-\text{distance}\left(u,v\right)}, \end{array}$$

(5) $$\begin{array}{c} {\text{sim}}_{d}\left(u,v\right)=\frac{\sum \left(p+\bar{p}\right)}{\sqrt{\left(p+\bar{p}\right)}}. \end{array}$$

ECM algorithm is a real-time online scanning algorithm for data streams, which can also be understood as a clustering algorithm for online data. The algorithm presets a real number threshold of cluster radius Dr, and based on the property that the distribution of data in the data stream changes over time, the ECM algorithm makes a clustering of the new data every time it enters the system. The ECM algorithm always controls the upper limit of the cluster radius utilizing a parameter threshold; that is, the cluster radius of a cluster stops growing when it increases to the value of Dr. Thus, the threshold value Dr controls the size of each clustering cluster by controlling the radius size and the size of each cluster, which affects the number of clusters and the clustering performance.

(6) $$\begin{array}{c} d\left(x,y\right)=\sqrt{\frac{\sum_{i=1}^{n}{\left(x-y_{i}\right)}^{2}}{q}}. \end{array}$$

In the clustering process, the data for the ECM algorithm originates from a continuous stream of online data. The ECM algorithm starts from an empty set and determines whether the data in the new data stream belongs to a currently existing cluster: if the new data belongs to an existing cluster, the cluster centre and the cluster radius of that cluster are updated; if the new data does not belong to any of the existing clusters, a new cluster is created. When a new cluster is created, the new data is used as the initial cluster centre of the new cluster, and the cluster radius *R* of the new cluster is initialized. The ECM algorithm dynamically increases the number of clusters, adjusts the cluster centres and the cluster radius in real-time regarding parameter thresholds, and may increase the cluster radius with each clustering, but when the cluster radius reaches the threshold, the cluster radius of the cluster is not updated. In modern technology, data streams have uncertainty in some aspects due to physical measurement limitations, interference from the surrounding environment, and other factors, such as frequent sexual instability or anomalies in some data streams [17]. The uncertainties contained in data streams can be divided into two categories: uncertainty of existence and uncertainty of attribute values. Therefore, the above two types of uncertainty based on uncertain data can usually be represented by statistics such as interval number or probability density function, and in this paper, multidimensional uncertain data streams are represented by interval numbers.

The ECM algorithm clusters deterministic data streams, and for achieving evolutionary clustering of multidimensional uncertain data, the ECM algorithm is not applicable. The MU-ECM algorithm uses the Euclidean distance between the data object and the centre of the clusters as the basis for determining the similarity between the data object and the clusters, and the smaller the distance, the greater the similarity. The smaller the distance value, the greater the similarity. The relationship between the distance value and the cluster radius is used as an important factor to determine whether the cluster radius is updated or not and whether the cluster centre is rediscovered or not, to obtain more accurate clustering results.

Also, clustering clusters may intersect with each other after formation because each cluster usually has an increasing cluster radius throughout the clustering process of the MU-ECM algorithm; that is, it is getting closer to the edges of other clusters in each dimension. As clustering continues, the increasing cluster radius also leads to larger intersection regions between neighbouring clusters. For example, triangles and circles represent samples in two different clusters, and their distributions are shown in Figure 2.

Although triangular objects and circular objects belong to two different clusters, there is an intersection of their edge points, and the objects within the intersection of the clusters are within the radius of both clusters. The intersection region is the similar region of two clusters and tends to expand continuously, which will make the number of data objects falling in the intersection region increasingly similar. Since different clusters have different sizes and different density fractions of objects within the clusters, the location distribution is also different, and it is not accurate to measure the similarity of two clusters by the distance between the centres of the two clusters or the distance of the closest samples. Therefore, the number of data objects in the cluster within the intersection range as a percentage of the total number of data objects in the cluster is used to characterize the degree of fusion to other clusters. The magnitude of the fusion degree indicates the degree of similarity between the most adjacent clusters of the cluster and can determine whether to fuse the two clusters. The clusters with high similarity can be selected for fusion, which ultimately ensures the accuracy of the final clustering results. Suppose that, for any cluster Ci, its fusion degree to any other cluster is calculated in the form shown in

(7) $$\begin{array}{c} \text{fus}\left(i,j\right)=\frac{h_{ij}}{h_{i}^{2}}. \end{array}$$

If the value of the shortest distance is less than the cluster radius value of the corresponding cluster, it is directly categorized; if the value of the shortest distance is greater than the cluster radius value of the corresponding cluster but close to some clusters, the corresponding cluster with the smallest difference between the distance value and the radius can be searched for to categorize. The data object is defined as the cluster centre of this cluster to create new clusters. Then, after getting multiple clusters, considering the possible intersection between clusters, the fusion degree between clusters is calculated and the degree of each fusion degree value is used to determine whether they should be fused into one cluster.

#### 2.1.2. Diagnostic Effect Experiment in Giant Cystic Tumour of the Oesophagus

All data were statistically analysed using SPSS 22.0 software. The correlates affecting recurrence metastasis and/or survival of GIST patients after preoperative imatinib adjuvant therapy were analysed using COX univariate and multifactorial analysis. The optimal threshold of pathological responsiveness after adjuvant therapy was investigated using ROC curves by maximizing the sum of sensitivity and specificity, minimizing the total error, and minimizing the distance between the cut-off value and the upper left corner of the ROC curve. The correlation between pathological responsiveness and each clinicopathological factor was analysed comparatively using the chi-square test. The Kaplan–Meier survival curve and log-rank method were used to analyse the relationship between tumour pathological responsiveness and recurrence-free survival and overall survival after adjuvant therapy [18]. The ROC curve actually represents a stochastic classifier. The faster the TPR grows and the larger the slope is, the better the classification performance of the model is reflected. The closer the ROC curve to the upper left corner, the higher the sensitivity and the lower the false positive rate. The point on the ROC curve closest to the upper left corner has the largest sum of sensitivity and specificity, and this point or its neighbouring points are often referred to as the diagnostic reference value. The recurrence-free survival time was calculated from the date of completion of surgery to the recurrence of surgical resection site or distant metastasis at other sites. Overall survival time was determined by counting the date of patient death from the date of completion of surgery. All statistical tests were two-sided in this paper, and a *p* value < 0.05 indicated a statistical difference.

Clinical symptoms of GIST patients may include gastrointestinal bleeding, obstruction, abdominal pain, and abdominal masses. GIST located in the oesophagus often shows symptoms of dysphagia, and malignant GIST may be accompanied by weight loss, liver metastases, abdominal implants, and so on. Some patients may come to the hospital for intestinal perforation [19]. The clinical symptoms of GIST patients are highly variable and lack their clinical specificity, and the symptoms are related to many factors, such as the location of the tumour, the size of the tumour, the malignancy of the tumour, and whether the tumour is ruptured or perforated. In the early stage of GIST, there may be no symptoms, and the symptoms appear relatively late, so it is not easy to attract the attention of the patients themselves. GIST tumours vary in size, and their clinical manifestations are variable and related to tumour size and location. Small tumours often have no clinical manifestations and are mostly detected during physical examination or laparotomy. The most common clinical symptom is gastrointestinal bleeding, which is caused by ulceration of the mucosal surface of the tumour, and patients present with vomiting blood, black stools, and anemia due to occult blood loss. Other symptoms include abdominal pain, abdominal masses, and debility. This may be accompanied by loss of appetite, fever, and weight loss. Frequent and scanty urination is seen in individual patients with rectal GIST. Individual cases with spontaneous rupture of the tumour and diffuse peritonitis as the first presentation have been reported. When the tumour diameter is relatively small, the first symptom is upper gastrointestinal bleeding, because the tumour diameter is small, but the mucosal surface often has ulcer formation, so there will be cystic necrosis, bleeding, and other manifestations, resulting in clinical symptoms of gastrointestinal bleeding. When the GIST tumour gradually increases and compresses the stomach and intestinal cavity, the symptoms of upper abdominal discomfort may appear, and when the tumour causes ulcers to form on the mucosal surface, the symptoms of peptic ulcer may appear. When GIST tumour ruptures, acute upper gastrointestinal bleeding symptoms may occur. When GIST has a long course, it may lead to weight loss, anemia, and other wasting symptoms, as shown in Figure 3.

Ultrasound endoscopy can better compensate for the shortcomings of general endoscopy and has the advantage of distinguishing the various layers of the gastric wall and the origin of the mass, that is, the specific layers and tissues of the gastric wall, as well as detecting exophytic GISTs that are difficult to detect by general endoscopy. GIST can be differentiated from other gastric tumours by ultrasound endoscopy, and if the tumour grows towards the lumen or mixed growth inside and outside the lumen, it can show displacement, separation, or even unfolding of the gastric mucosa due to compression, and at the same time, barium radiography can indicate destruction of the mucosa of the gastric wall, filling defect, disorder or even ulcer formation, and so on; however, barium radiography also has its drawbacks. However, barium radiography also has the drawback that it is difficult to diagnose GIST with extraluminal growth, and therefore the diagnostic rate is not high. This ancillary test was not used in the present study.

The tumour diameter of gastric mesenchymal tumour and small intestinal mesenchymal tumour can be compared by the chi-square test, and the tumour diameter of gastric mesenchymal tumour is smaller, while the tumour diameter of small intestinal mesenchymal tumour is larger. In contrast, small intestinal mesenchymal tumours with a small diameter or obvious clinical symptoms are often difficult to be detected. Meanwhile, when comparing the postoperative NIH risk ratings of gastric mesenchymal tumour and small intestinal mesenchymal tumour, 38 patients with gastric mesenchymal tumour were at very low risk, 31 patients at low risk, 32 patients at intermediate risk, and 19 patients at high risk, while 3 patients with small intestinal mesenchymal tumour were at very low risk, 8 patients at low risk, 4 patients at intermediate risk, and 20 patients at high risk. By comparing the risk classification results of both, it can be found that small intestinal mesenchymal tumour has a higher risk compared with gastric mesenchymal tumour, as shown in Figure 4.

Therefore, it is necessary to distinguish between the priority of evil and deficiency and to choose the priority and sequence of treatment to support and eliminate evil. This is the key to improve the efficacy of difficult diseases; from the pathogenesis, we can also see that such patients often have damp-heat or cold-heat mismatch, and the treatment should be warming and clearing [20]. Among them, there were 53 patients with very low risk, 42 patients with low risk, 42 patients with medium risk, and 65 patients with high risk. A total of 69 high-risk patients were followed up, among whom 26 patients were taking imatinib adjuvant therapy after surgery, with a dosing rate of 37.68%. In comparison with other studies with larger sample sizes, the postoperative imatinib dosing rate in patients with intermediate to high risk was 60.47%, 68.35%, 49.06%, and 52.86%, respectively. The reason for the low rate of postoperative imatinib in the high-risk patients in this study may be related to the poor economic conditions of patients in the region and their inability to afford the drug. Gastrointestinal lesions occurring in combination with small GIST were predominantly malignant, mostly carcinomas, including adenocarcinoma, and squamous cell carcinoma, with high to moderate differentiation in squamous cell carcinoma and moderate to low differentiation in adenocarcinoma, which is generally consistent with the literature [21]. One case of oesophageal carcinoma was a mixed squamous cell carcinoma and small cell carcinoma, and the other was a basal cell-like squamous cell carcinoma; in addition, other rare types were lymphoma (MALT lymphoma in this group, which was also combined with a hyperplastic polyp of the appendix in this case) and squamous epithelial atypical hyperplasia, the latter two being rarely reported combined tumours. The benign tumours were juvenile polyps and hyperplastic polyps, which were also rarely reported. The benign tumours are juvenile polyps and hyperplastic polyps which are also rarely reported. The onset of the disease is mainly concentrated in the stomach and oesophagus. Treatment is based on digestive system lesions, especially in cases with combined digestive system cancer. Tumour compression symptoms are commonly found in the intracranial, cervical, mediastinal, retroperitoneal, and intravertebral canal. For example, intracranial tumours compressing the brain parenchyma cause increased intracranial pressure, which may cause headache, nausea, vomiting, and visual disturbance. The tumour of the thyroid gland may press the laryngeal nerve and cause hoarseness. If it presses on the trachea or esophagus, it causes difficulty in breathing or swallowing.

### 2.2. Analysis of Results

#### 2.2.1. Algorithm Performance Analysis

In the experimental process, to observe the influence of the different proportion of similarity of user attributes and similarity of ratings and category preferences on the experimental results, the parameter values of *r* and *ω* were adjusted continuously during the experimental process, the value of *k* was also adjusted continuously to select the optimal nearest neighbours, and the final experimental results were compared and analysed with the traditional correlation algorithm after parameter tuning. The experimental results are shown in Figure 5, which shows that the MAE value is the lowest when the *R*-value is 0.9 and the experimental results are the best.

Different items have different attribute characteristics, which will affect the size of the final user rating to a certain extent. The existing data set has high-dimensional item attributes, so we first introduce PCA technology to reduce the dimensionality of the item attribute data and do the calculation of item similarity based on the reduced dimensional attribute data. Secondly, the item similarity is fused with the WSO algorithm for prepopulation of ratings, and then the user rating similarity is further calculated. In addition to tumour size, the primary site and the number of nuclear schwannomas are also key factors in determining the prognosis of the disease. The NIH subsequently developed a standard for assessing the malignancy of gastrointestinal mesenchymal tumours by combining tumour size and the number of nuclear schwannomas and assessed the malignancy of this tumour by the risk of invasion, which is classified into four grades: very low, low, moderate, and high risk of invasion. Currently, the common grading diagnosis for gastrointestinal mesenchymal tumours is the NIH criteria. The WSO algorithm uses the number of users who jointly rates the items as the corresponding weights for the weighted rating prediction but does not consider the effect of interitem similarity on user rating differences. Taking movies as an example, most female friends like literary and family movies, while they have a low preference for war crime movies, so when these two types of movies are rated together, there is a large difference in ratings.

As can be seen from Figure 6, the average running time of the MU-SAECM algorithm in the test dataset is significantly lower than that of the other four algorithms, and the variation is relatively small. This is because in the later clustering of the data, along with the increase of the cluster radius, the distance between the data object and the cluster centre is increasingly likely to be smaller than the cluster radius, so it is increasingly likely that it can be directly classified into the clusters. The MU-SAECM algorithm also uses the number of intervals and distance calculation to represent the uncertainty of the data, which avoids the problem of large computation caused by the integral operation and improves the algorithm's efficiency. In contrast, the UIDMicro algorithm has a large impact on the number of members' threshold, which makes the clustering model update with a large delay or too frequent clustering update; the EDMicro algorithm requires more iterative steps, which requires more time overhead to update the microcluster structure in the form of MBR in each step. The MU-ECM algorithm and the ECM algorithm require multiple accesses to the historical data in one execution. The MU-ECM algorithm and the ECM algorithm require multiple accesses to historical data at one time, and the efficiency of the ECM algorithm is susceptible to the threshold value as the number of data increases. The time advantage of the MU-SAECM algorithm over the other four algorithms becomes increasingly obvious when the number of uncertain data becomes larger.

The MU-SAECM algorithm has improved the clustering efficiency by incorporating feature triples while making the clustering of interval-type data closely related to its characteristics. It is suitable for clustering analysis of data streams, and the new computational form of interval-type data combines two elements of intervals simultaneously, which can reflect the influence of uncertainties in the clustering results. The MU-SAECM algorithm is proposed to solve the clustering problem in multidimensional uncertain data streams. The representation of the interval number is improved so that the algorithm is highly adaptive to the interval width, and a new formula combining the interval number and the Euclidean distance formula is used as a new calculation method to calculate the spacing between clusters and between clusters and data elements. Also on data object categorization, the interval number and distance calculation are combined to propose a new method of similarity categorization based on Euclidean distance. In the case that intersection may be generated between multiple clusters generated by preclustering, the fusion of two clusters with greater similarity is realized at the same time to prevent the case that cluster fusion is excessive to generate only one cluster. The idea of internal partitioning of clusters using density clustering is proposed to ensure the reliability of clustering results.

#### 2.2.2. Diagnostic Effect Results

Gastroscopy and ultrasound endoscopy are common tests for gastric mesenchymal tumours and are valuable in the diagnosis of mesenchymal tumours and in helping to assess the risk of malignancy of the lesion. Data clustering, on the other hand, analyses and divides data that would otherwise have no category reference into different groups, that is, derives class labels from these data. Cluster analysis itself is to discover information about data objects and their relationships based on the data and to group these data. The objects within each group are similar to each other, while the objects between the groups are unrelated. It is easy to understand that the higher the similarity within groups and the higher the dissimilarity between groups, the better the clustering. Gastric mesenchymal tumours appear gastroscopically as hemispherical, fusiform, or irregularly shaped submucosal masses with a smooth surface mucosa, sometimes with erosions, ulcers, and bleeding. EUS is the most used tool to identify submucosal masses in the GI tract by scanning the wall of the GI tract with a miniature high-frequency ultrasound probe mounted on top of the endoscope, which can clearly show the level and echogenicity of the wall. The first, third, and fifth layers are high echogenic bands, which correspond to the superficial mucosal layer, submucosal layer, and plasma layer, while the second and fourth layers are low echogenic bands, which correspond to the mucosal muscle layer and intrinsic muscle layer. As a basis for determining the likelihood of tumour recurrence after surgery and predicting treatment outcome and prognosis, positive circumferential margins, presence of vascular infiltration and perineural infiltration, poor response to neoadjuvant therapy, BRAF gene mutation, and microsatellite stability can be considered as indicators of high recurrence rate and poor prognosis, which also indicate the need for more aggressive and comprehensive adjuvant therapy after surgery. Gastric mesenchymal tumours appear endoscopically as hypoechoic homogeneous masses, which may be accompanied by punctate hyperechoic and cystic echogenicity, most of which originate from the lamina propria and a few from the submucosa. Smooth leiomyosarcoma appears as a round or oval hypoechoic endoscopic mass with clear borders, originating from layer 2 or layer 4 of the gastric wall. Ectopic pancreatic echogenic endoscopy showed hypoechoic or mixed echogenicity, sometimes with tubular structures, and could originate from layers 2–5 of the gastric wall, as shown in Figure 7.

In a large sample size study, CD117 expression was detected in 985 of 1040 GIST patients, representing an expression rate of approximately 94.7%. In addition, CD117 is barely expressed in smooth muscle tumours, smooth muscle sarcomas, nerve sheath tumours, etc., suggesting that CD117 is indeed a highly sensitive and specific marker for GIST, as shown in Figure 8.

For the evaluation of pathological response after preoperative adjuvant therapy for tumours, TRG aims to grade the pathological response of tumours after adjuvant therapy and to assess the effect of patients on preoperative adjuvant therapy and has been applied to rectal cancer, oesophageal cancer, and gastric cancer. In contrast, PCR is still more often used in clinical practice with a focus on PCR because it can ensure the prognostic safety of patient survival and is also following relevant ethical norms. In our study, the pathological response after adjuvant therapy was taken as a threshold of 40%, which can accurately distinguish the prognosis of patients. We believe that the effectiveness of imatinib treatment varies among patients, that patients with a pathological response of >40% after imatinib treatment have a better prognosis, and that such patients are more effective for imatinib adjuvant therapy, which is important for guiding individualized treatment after surgery.

## 3. Conclusion

Firstly, an evolutionary clustering algorithm for clustering multidimensional uncertain data streams is proposed: the MU-ECM algorithm. Then, we improve the Euclidean distance calculation method in the ECM algorithm to consider the information of each dimension when dealing with multidimensional data, so that we can find the clear degree of similarity between data objects. This rule does not need to rely on predefined thresholds as in the ECM algorithm and avoids the situation that thresholds affect the final clustering results. The present study did not compare microwave ablation with other thermal ablation techniques (e.g., radiofrequency ablation), and the efficacy of microwave ablation in clinical practice can be further demonstrated in a controlled trial. Due to the limitations, the pathological evaluation in this study could also be more convincing if the material was punctured from each patient at each time point for its control.

## Figures and Tables

**Figure 1:** Framework of EUS-RTE algorithm for clustering analysis.

**Figure 2:** Two clusters with a certain similarity.

**Figure 3:** Diagnostic features.

**Figure 4:** Relationship between symptoms.

**Figure 5:** Effect of *R*-value on MAE.

**Figure 6:** Running time of the five algorithms with different data sets.

**Figure 7:** Functional changes at different times.

**Figure 8:** Comparison of patient outcomes in different groups.

## Data Availability

The data used to support the findings of this study are available from the corresponding author upon request.
